This article has been retracted.

# A Case-Control Study of Photodynamic Therapy Combined with Thymosin in the Treatment of Condyloma Acuminatum in Anal Canal

**DOI:** 10.1155/2022/3019379

**Published:** 2022-03-12

**Authors:** Xia Qing Wang, Yi Hu, Ke Hong

**Affiliations:** ^1^Department of Dermatology and Venereology, The Eighth Hospital of Wuhan, Wuhan 43000, China; ^2^Department of Infectious Diseases, Wuhan Jinyintan Hospital, Wuhan 43000, China

## Abstract

A case-control study is performed in this paper to explore various possible effects and clinical value of the photodynamic therapy combined with thymosin for the treatment process of the condyloma acuminatum (CA) in the anal canal. For this purpose, a hundred (100) patients specifically with CA in the anal canal who were regularly treated in the hospital from February 2019 to April 2021 were recruited. The first group, that is, the control group, was treated with thymosin, whereas photodynamic therapy combined with thymosin was used as a treatment for the study group. The curative effect, clinical index, LTN, SP, TGF-*β* 1, TNF-*α*, CD3+, CD4+, CD8+, and the adverse reactions of incidence were compared between these groups. Moreover, 27 cases were observed to be obviously effective, 22 were observed to be effective, and a single case was observed to be ineffective. Thus, 98% is the total effective rate where a single case relapses. Likewise, in the control group, 15 cases were observed to be obviously effective, 28 effective, and 13 ineffective. Thus, 86% is the total rate of effectiveness where thirteen (13) cases relapse. We have observed that the study group has a higher rate of effectiveness than the control group and the rate of recurrence of the former group was slightly lower than that of the latter group, that is, the control group (*P* < 0.05). In addition, the time of symptom improvement, the amount of bleeding, the disappearance time of bloody stool, and the time of the first recurrence of the study group were observed to be lower than those of the control group (*P* < 0.05). In levels of LTN and SP, we have observed no or zero significant differences between these groups before treatment. However, LTN's levels of both groups increased after the treatment, and SP's level decreased. LTN's level of the study group was observed to be higher than that of the other group, and SP's level in the former group was lower than that in the latter group. Zero significant differences were observed in the TGF-*β* 1 and TNF-*α*'s levels between these groups before treatment, but the level of TGF-*β* 1 and TNF-*α* has increased and decreased, respectively, in both groups specifically after treatment. The level of TGF-*β* 1 in the former group was observed to be slightly higher than that in the latter group, that is, the control group, while TNF-*α*'s level in the study group was lower than that in the control group. We have not observed any significant difference in CD4+, CD3+, and CD8+ levels between these groups before treatment. However, after treatment, CD3+ and CD4+ levels increased, and the levels of CD8+ decreased in both groups, while CD3+ and CD4+ levels in the former group were evident to be higher than those in the latter group and the level of the CD8+ in the study group was observed to be lower than that in the control group. Finally, we compared the adverse reactions of incidence between these groups. There were 4 cases of tingling sensation and 1 case of redness and swelling in the group study along with a total incidence of 10%. There were 5 cases of tingling sensation and 2 cases of redness and swelling in the control group along with a total incidence of 14%. The incidence of adverse reactions in the study group was observed to be slightly lower than that in the control group, but a significant difference was not observed between these groups (*χ*^2^ = 0.378; *P* > 0.05).

## 1. Introduction

Condyloma acuminatum (CA) is a common sexually transmitted disease, which is mainly transmitted through sexual contact. At present, there are many ways to treat CA, but the recurrence rate is still high [1]. We found that perianal infection accounted for more than 1/4 of all infected patients by clinical research. Male infection was 6 times that of women, so the incidence rate of anal CA was not neglecting [2, 3]. The pathogen of CA is human papillomavirus (HPV); more than 100 types of HPV have been identified, of which about 30 are related to the occurrence of CA. CA in the anal canal is prone to be missed due to its concealed location, difficult exposure, and no obvious symptoms. The treatment of CA in the anal canal has a narrow field of vision, and it is easy to hide dirt in the anal canal. No matter it is a laser, electric burn, or drug infusion, it cannot avoid the disadvantages of repeated and repeated treatment [4]. The common treatments of CA include CO2 laser, cryotherapy, surgical resection, electroresection, and curettage and can also be combined with immunoregulatory drugs such as Zhenqi Fuzheng capsule, but considering that it can only remove the lesions visible to the naked eye, the latently infected keratinocytes still exist, so that the above treatment is effective in a short time, but the recurrence rate is high [5, 6]. The important causes of recurrence are the presence of subclinical infection around warts and different degrees of low or abnormal cellular immune function in the patients. Clinical studies have shown that CA recurrence factors are complex, mainly related to skin damage that has not been thoroughly cleaned up and HPV potential infection [7, 8]. Photodynamic therapy is mainly 5-aminolevulinic acid, which is a new method widely used at present, which is effective for subclinical infection and potential infection, but the effect of single use is not good for patients with large warts [9].

In this paper, a case-control study is performed to explore various possible effects and clinical value of the therapy of the photodynamic combined with thymosin for the treatment process of the condyloma acuminatum (CA) in the anal canal. For this purpose, a hundred (100) patients specifically with CA in the anal canal who were regularly treated in the hospital from February 2019 to April 2021 were recruited. The first group, that is, the control group, was treated with thymosin, whereas photodynamic therapy combined with thymosin was used as a treatment for the study group. The curative effect, clinical index, LTN, SP, TGF-*β* 1, TNF-*α*, CD3+, CD4+, CD8+, and the adverse reactions of incidence were compared between these groups. Moreover, 27 cases were observed to be obviously effective, 22 were observed to be effective, and a single case was observed to be ineffective. Thus, 98% is the total effective rate where a single case relapses. Likewise, in the control group, 15 cases were observed to be obviously effective, 28 effective, and 13 ineffective. Thus, 86% is the total rate of effectiveness where thirteen (13) cases relapse. We have observed that the study group has a higher rate of effectiveness than the control group and the rate of recurrence of the former group was slightly lower than that in the latter group, that is, the control group (*P* < 0.05). In addition, the time of symptom improvement, the amount of bleeding, the disappearance time of bloody stool, and the time of the first recurrence of the study group were observed to be lower than those of the control group (*P* < 0.05). In levels of LTN and SP, we have observed no or zero significant differences between these groups before treatment. However, LTN's levels of both groups increased after the treatment, and SP's level decreased. LTN's level of the study group was observed to be higher than that of the other group, and SP's level in the former group was lower than that in the latter group. Zero significant differences were observed in the TGF-*β* 1 and TNF-*α*'s levels between these groups before treatment, but the level of TGF-*β* 1 and TNF-*α* has increased and decreased, respectively, in both groups specifically after treatment.

The rest of the paper has been arranged as follows.

In Section 2, the proposed evaluation method along with generalized information on the selection and rejection criterion for the experimental setup is presented, which is followed by a comparative analysis section of the various experimental results and observations. A generalized discussion section is provided, which is followed by a comprehensive section on the concluding remarks.

## 2. Proposed Methodology: Patients and Method

### 2.1. General Information

Hundred (100) patients, preferably having CA in the anal canal, were treated in the hospital, specifically from February 2019 to April 2021. These patients were divided through a random procedure into two groups, that is, control and study. In the control group, the age was 18–45 years, the average age was 30.37 ± 3.55 years, including 34 males and 16 females, the course of disease ranged from 1 to 7 months, the average course of the disease was 3.85 ± 1.85 months, the size of warts was 2–8 cm, and the average size of warts was 5.38 ± 1.85 cm. In the study group, the age was 18–46 years, the average age was 30.86 ± 3.75 years, including 35 males and 15 females, the course of the disease was 1–7 months, the average course of the disease was 3.86 ± 1.62 months, the size of warts was 2–8 cm, and the average size of warts was 5.75 ± 1.81 cm. There was no statistical significance in the general data of the two groups. This study was approved by the Medical Ethics Association of the hospital, and every patient willingly signed the consent.

The inclusion criteria were as follows: acute dampness in the anal canal was diagnosed by clinical and pathological examination, which was the first onset, and no antiviral treatment was taken.

The exclusion criteria were as follows:

1. Patients with incomplete general medical records.
2. Patients having severe renal and hepatic dysfunction.
3. Patients with immune diseases and other infectious diseases.
4. Women during pregnancy and lactation.
5. Those who are allergic or intolerant to thymosin enteric tablets.
6. Those who cannot tolerate photodynamic therapy.

### 2.2. Proposed Technique

The control group received oral thymopeptide enteric-coated tablets (H20058365; Heilongjiang Dilong Pharmaceutical Co., Ltd.; specification: 20 mg), 20 mg, 3 times a day for 30 days. The treatment method of thymosin in the study group was the same as that in the control group. 5-aminolevulinic acid photodynamic therapy (ALA-PDT) was performed using a solution with a concentration of 20%, evenly smeared on the affected area of the wart and the surrounding skin 2 cm while using aseptic plastic wrap. After 3.5 hours of encapsulation, the aseptic plastic capsule was removed and irradiated with photodynamic therapy apparatus. The affected area was irradiated for 15–20 min with an energy density of 100 J/cm^2^, wavelength of 635 nm, and irradiation distance of 5 cm/10 cm once a week for 30 days.

### 2.3. Observation Indicators

#### 2.3.1. Curative Effect Evaluation

1. Make a diagnosis with reference to the “Standard for Diagnosis and Treatment of Condyloma Acuminatum (trial)” compiled by the Ministry of Health in 2000. Significant effect: the follow-up for 6 months after treatment showed that there was no new skin lesion and no verrucous body recurrence, and wound healing was good; effective: after treatment, the wart body decreased significantly, and the wound healed well; ineffective: the wart body of the patient did not decrease or even increase after treatment; recurrence: the original site of the patient appeared new skin shun or wart body after treatment. Total effective rate = effective + obviously effective rates.
2. The clinical indexes of symptom improvement time, bleeding volume, disappearance time of bloody stool, and first recurrence time were observed in the two groups.

#### 2.3.2. LTN, SP, TGF-*β*1, TNF-*α*, and Detection Methods of CD3+, CD4+, and CD8+ Levels

1. The levels of cellular chemokine (LTN) and TNF-*α* were detected. We performed the following: labeling the enzyme plate at room temperature, preparing the standard sample, diluting the sample, adding 100 *μ*l/well serum and standard sample to each well, wet incubating at 37°C for 2 hours, washing the reaction plate repeatedly, adding 100 *µ*l/well antibody working solution according to 1 *μ*l/well, wetting 45 min twice, washing reaction plate, adding 100 *µ*l/well TNF-*α* and LTN solution per well, wet incubation 45 min, and adding 100 *µl*/well termination solution to terminate the reaction. The wavelength of 450 nm was measured, and the level of factor to be measured was calculated.
2. Changes of SP level before and after treatment: venous blood 6 ml was taken from patients before and after treatment, 20 min was centrifuged under 2000 r/min, and the upper serum solution was separated statically and kept for detection at −80°C. The blood was injected into a precooled test tube containing disodium 0.5 mol/L ethylenediamine tetraacetate and an aprotinin tube containing 40 *µl* aprotinin. The blood was centrifuged 15 min at 4°C and 3000 r/min and preserved in plasma at −20°C. The level of SP was detected by radioimmunoassay, and the operation was carried out in strict accordance with the steps described in the SP kit.
3. The levels of CD3+, CD4+, and CD8+ before and after treatment: the level of T lymphocyte subsets was detected by indirect method. The fasting venous blood 5 ml to be tested was passed on to a 5-well plate, cultured in saturated humidity of 37°C and 5% carbon dioxide for 3 days, then digested with 0.25% trypsin, and centrifuged 5 min under 2000 r/min; cells were collected and repeatedly washed with PBS buffer after collection; again cells were collected after centrifugation and propidium iodide staining solution 1 ml was added. After being kept away from light at 36–37.2°C for 1 h, PE fluorescence staining was used for specific fluorescence labeling. Photons were emitted during the flow under the sheath fluid, and the levels of CD3+, CD4+, and CD8+ were detected strictly according to flow cytometry.
4. Detection of TGF-*β* 1 level: the level of TGF-*β* 1 was detected by SP immunohistochemical staining. The tested samples were treated with dewaxing and hydration, soaked in citrate buffer at 0.01 mol/L and 95°C, and hot repaired. After 10 years of culture, in the environment of 3% H2O2, we dropped goat serum, let it stand for 30 minutes, cultured it at 26 °C for 30 minutes, then extracted the sealing solution, added the first antibody, and cultured it overnight at 5 °C, we added the second antibody, and finally let it stand for 30 minutes and cultured it in the incubator at 37 °C. After cleaning, DAB was used to develop color and seal the film.

#### 2.3.3. Incidence of Adverse Reactions

In these groups, adverse reaction incidence was computed.

### 2.4. Statistical Analysis

To verify the proposed scheme's performance, we have utilized SPSS21.0, which is a statistical tool, to extensively examine the proposed scheme. Data measurements were represented in the form of $\bar{x}$ ± *s*. Prior to the statistical analysis, homogeneity of variance and normal distribution were tested along with a *t*-test that is utilized for the comparison of these groups. All counting data were represented as *n* (%), and the *χ*^2^ test was used for statistical analysis. Finally, we have observed a statistically significant difference (*P* < 0.05).

## 3. Experimental Results and Evaluation

### 3.1. Comparison of Clinical Efficacy

The study group consisted of 27 obviously effective cases, 22 effective cases, and 1 ineffective case, whereas the total rate of effectiveness was 98%, of which only 1 case relapsed, while in the control group, 15 obviously effective, 28 effective, and 13 ineffective cases were present, whereas the total rate of effectiveness was 86%, of which 13 cases relapsed. The total rate of effectiveness of the former group was higher than that of the latter group, whereas the rate of recurrence is inverse; that is, the latter group has a higher value. We have observed a difference that was significant statistically between these groups (*P* < 0.05). All the data were presented in Table 1.

### 3.2. Comparison of Symptom Improvement Time, Bleeding Volume, Disappearance Time of Bloody Stool, and First Recurrence Time

The time of symptom improvement, the amount of bleeding, the time of disappearance of bloody stool, and the first recurrence time in the former group were lower than those in the latter group, whereas data were observed to be significant, that is, statistically (*P* < 0.05). All the data were presented in Table 2.

### 3.3. Time of First Recurrence

In terms of LTN and SP horizontal before treatment, we have not observed any difference, which was significant, between these groups (*P* ＞ 0.05). After treatment, LTN's level increased in these groups, whereas SP's levels decreased. The level of LTN in the study group was higher than that in the control group, while the level of SP was lower than that in the control group (*P* ＜ 0.05). All the data were presented in Table 3.

### 3.4. TGF-*β*1 and TNF-*α*

In terms of TGF-*β*1 and TNF-*α*, before treatment, we have not observed any significant difference between these groups (*P* > 0.05); after treatment, TGF-*β*1's level in these groups has increased, whereas TNF-*α*′s levels have decreased. TGF-*β*1's levels in the former group were higher than those in the latter group, while TNF-*α*′s levels in the former group were lower than those in the latter group. All the data were presented in Table 4.

### 3.5. CD3＋, CD4＋, and CD8＋

We have not observed any significant difference in CD8+, CD4+, and CD3+ levels between these groups, particularly before treatment, but the levels of CD4+ and CD3+ increased, and the level of CD8+ decreased in both groups after treatment. The levels of CD3+ and CD4+ in the former group were slightly higher than those in the latter group, while the level of CD8+ in the former group was lower than that in the latter group. All the data were presented in Table 5.

### 3.6. Comparison of the Incidence of Adverse Reactions

Comparing the incidence of adverse reactions between the two groups, there were 4 cases of tingling sensation and 1 case of redness and swelling in the study group, with a total incidence of 10%, while in the control group, there were 5 cases of tingling sensation and 2 cases of redness and swelling, with a total incidence of 14%. The adverse reaction incidence in the former group was observed to be lower than that in the latter group. However, zero significance differences were observed between these groups (*χ*^2^ = 0.378; *P* > 0.05).

## 4. Discussion

CA remains a sexually transmitted disease induced by human papillomavirus (HPV) infection. The incidence of CA is 3 times higher than that of genital herpes, and CA is closely linked with the occurrence of genital cancer [10]. The main clinical symptom of CA is the proliferative injury of the anus and genitalia caused by HPV infection, which is in the shape of cauliflower or thorn. For CA, the incubation period ranges from three weeks to eight months, whereas the average period is approximately three months [11, 12]. The incidence of CA is mainly in young people aged 20 to 30 years [13]. During the onset of CA, most cases have no symptoms, and some cases can be accompanied by pain and ulcer bleeding and even cause genital cancer [14]. CA has the characteristics of strong infectivity, easy recurrence, and difficult to cure, which has a serious impact on the quality of life of patients. The polypeptide hormone produced by thymic epithelial cells is called thymosin, which is an immunomodulator and is used in the treatment of CA by inducing T cell differentiation and regulating immune balance. Compared with thymosin injection, oral preparation has the advantages of good compliance and easy to take and carry, and the degree of acceptance of patients is higher [15–17]. Photodynamic therapy utilizes molecular oxygen induced by photosensitizer and light source to selectively break the ring of target tissue cells with 5-aminolevulinic acid. The second-generation photosensitizer is not photosensitive. It metabolizes with the heme synthesis pathway into active photosensitizer protoporphyrin IX to produce photosensitivity. Reactive oxygen species are produced after irradiation at specific wavelengths to kill proliferative and active cells, resulting in slight damage to the surrounding normal tissue. In terms of absorptivity and penetration depth, the red light of 635 nm is the most commonly used clinical light source. At present, LED light source is widely used [18–20].

At present, three-stage therapy is commonly recommended for the treatment of CA in the anal canal in China. The first step is to remove warts visible to the naked eye, the second step is to use Ella-photodynamic therapy to remove the warts of subclinical infection and latent infection, and the third step is to consolidate the treatment and improve the immune level [21, 22]. After Rao Lang et al. used this method to treat CA in the anal canal, all patients had pain during defecation and blood in the stool. The authors analyzed that the above adverse reactions were related to the traditional carbon dioxide laser treatment in the first step [23]. The first group, that is, the control group, was treated with thymosin, whereas photodynamic therapy combined with thymosin was used as a treatment for the study group. The curative effect, clinical index, LTN, SP, TGF-*β* 1, TNF-*α*, CD3+, CD4+, CD8+, and the adverse reactions of incidence were compared between these groups. Moreover, 27 cases were observed to be obviously effective, 22 were observed to be effective, and a single case was observed to be ineffective. Thus, 98% is the total effective rate where a single case relapses. Likewise, in the control group, 15 cases were observed to be obviously effective, 28 effective, and 13 ineffective. Thus, 86% is the total rate of effectiveness where thirteen (13) cases relapse. We have observed that the study group has a higher rate of effectiveness than the control group and the rate of recurrence of the former group was slightly lower than the latter group, that is, the control group (*P* < 0.05). Of note, the symptom improvement time, bleeding volume, blood stool disappearance time, blood stool disappearance time, and first recurrence time in the study group were lower than those in the control group. Comparing the incidence of adverse reactions between the two groups, there were 4 cases of tingling sensation and 1 case of redness and swelling in the study group, with a total incidence of 10%, while in the control group, there were 5 cases of tingling sensation and 2 cases of redness and swelling, with a total incidence of 14%. The incidence of adverse reactions in the study group was lower than that in the control group, but there was no significant difference between the two groups. Our study demonstrated that thymosin combined with photodynamic therapy effectively reduced the number and area of CA in the anal canal and reduced the adverse reactions caused by drugs, while the tingling, redness, and swelling occurred during the treatment.

Related research results show that LTN, SP, and other immune factors are closely related to the occurrence, development, and recurrence of CA [24]. LTN can effectively attract leukocytes to gather in the infected site and participate in the regulation of immune function by activating natural killer cells, T cells, and enhancing mucosal immunity. As a neuropeptide is related to pain transmission, SP participates in immune activities. Related research results show that SP uses *G* protein-coupled receptors to accelerate the mitosis of infected HPV cells and promote the growth of wart tissue, thus affecting the occurrence and development of CA[24]. Combined with the results of this study, there was no significant difference in the levels of LTN and SP between the two groups before treatment. After treatment, the level of LTN in both groups increased, and the level of SP decreased. The level of LTN in the study group (288.76 ± 28.86 pg/ml) was higher than that in the control group (265.91 ± 28.96 pg/ml), and the level of SP (54.91 ± 6.91 ng/L) was lower than that in the control group (65.91 ± 10.31 ng/L). TGF-*β*1, derived from keratinocytes and fibroblasts, is a member of the transforming growth factor family, which can effectively inhibit epithelial cell proliferation, regulate immunity, and effectively regulate cell growth, differentiation, and apoptosis [25]. High expression of TNF-*α* can produce a cytotoxic response to T cells and enhance inflammatory response so as to achieve the inhibition of immune function, destroy the balance between anti-inflammatory response and proinflammatory response, and lead to repeated attacks of condyloma acuminatum [25]. Our results showed that, after photodynamic therapy combined with thymosin enteric-coated tablets, the level of TGF-*β*1 increased and the level of TNF-*α* decreased in both groups. The level of TGF-*β* 1 in the study group (11.56 ± 1.91 ng/ml) was higher than that in the control group (125.93 ± 19.85 ng/L). The level of TNF-*α* in the control group was lower than that in the control group (196.92 ± 23.85 ng/L).

There are two main effects of cellular immunity: the first is specific binding of target cells, destruction of the target cell membrane, and direct killing of target cells; the other is the release of lymphokines, which eventually expand and enhance the immune effect [26]. T lymphocytes account for about 65% of the total lymphocytes in peripheral blood, accounting for 75% of the total lymphocytes and up to more than 95% in the chest catheter. Cytotoxic T cells destroy infected cells, which function as a killer or cytotoxin because they can kill target cells that produce a special anti-inflammatory response. The main surface marker of cytotoxic T cells is CD8, also known as killer T cells [26]. In this study, there was no significant difference in the levels of CD3+, CD4+, and CD8+ between the two groups before treatment. After treatment, the levels of CD3+ and CD4+ in both groups increased, and the levels of CD8+ decreased. The levels of CD3+ and CD4+ in the study group were higher than those in the control group (CD3+, 51.85 ± 2.91%; CD4+, 35.96 ± 1.56%, resp.). The level of CD8+ in the study group was lower than that in the control group (34.81 ± 2.34%). Related studies have shown that the levels of CD3+, CD4+, and CD8+ in peripheral hematoma of patients with condyloma acuminatum in the anal canal are significantly lower than those without recurrence, indicating that there is a significant correlation between the recurrence rate of patients with condyloma acuminatum in the anal canal and their own immune level [27]. The determination of the levels of CD3+, CD4+, and CD8+ in patients with CA in the anal canal is of great clinical significance to evaluate the prognosis and observe the curative effect. CD4+ enhances the immune response by secreting cytokines, while CD8+ suppresses the immune response by secreting inhibitory factors or by itself.

## 5. Conclusion

In this paper, a case-control study is performed to explore various possible effects and clinical value of the therapy of the photodynamic combined with thymosin for the treatment process of the condyloma acuminatum (CA) in the anal canal. For this purpose, a hundred (100) patients specifically with CA in the anal canal who were regularly treated in the hospital from February 2019 to April 2021 were recruited. The first group, that is, the control group, was treated with thymosin, whereas photodynamic therapy combined with thymosin was used as a treatment for the study group. The curative effect, clinical index, LTN, SP, TGF-*β* 1, TNF-*α*, CD3+, CD4+, CD8+, and the adverse reactions of incidence were compared between these groups. Moreover, 27 cases were observed to be obviously effective, 22 were observed to be effective, and a single case was observed to be ineffective. Thus, 98% is the total effective rate where a single case relapses. Likewise, in the control group, 15 cases were observed to be obviously effective, 28 effective, and 13 ineffective. Thus, 86% is the total rate of effectiveness where thirteen (13) cases relapse. We have observed that the study group has a higher rate of effectiveness than the control group and the rate of recurrence of the former group was slightly lower than the latter group, that is, the control group (*P* < 0.05). In addition, the time of symptom improvement, the amount of bleeding, the disappearance time of bloody stool, and the time of the first recurrence of the study group were observed to be lower than those of the control group (*P* < 0.05). In levels of LTN and SP, we have observed no or zero significant differences between these groups before treatment. However, LTN's levels of both groups increased after the treatment, and SP's level decreased. LTN's level of the study group was observed to be higher than that of the other group, and SP's level in the former group was lower than that in the latter group. Zero significant differences were observed in the TGF-*β* 1 and TNF-*α*'s levels between these groups before treatment, but the level of TGF-*β* 1 and TNF-*α* has increased and decreased, respectively, in both groups, specifically after treatment. Meanwhile, photodynamic therapy combined with thymosin can improve the therapeutic effect, reduce the recurrence rate, provide high safety, and provide a theoretical basis for the clinical treatment of CA in the anal canal.

## Figures and Tables

**Table 1:** Control versus study groups: clinical efficacy (*n*/%).

Group	Cases	Significance	Effective	Invalid	Relapse	Total efficiency
Control group	50	15 (30.00)	28 (56.00)	7 (14.00)	13 (26.00)	43 (86.00)
Study group	50	27 (54.00)	22 (44.00)	1 (2.00)	1 (2.00)	49 (98.00)
*χ* ^*2*^					11.961	4.891
*P*					0.000	0.026

**Table 2:** Comparison of symptom improvement time, bleeding volume, disappearance time of bloody stool, and first recurrence time (*x* ± *s*).

Group	Cases	Symptom improvement time (d)	Bleeding volume (ml)	Time of disappearance of blood stool (d)	Time of first recurrence (d)
Control group	50	6.04 ± 1.22	34.85 ± 3.91	1.95 ± 0.21	10.82 ± 3.91
Study group	50	3.95 ± 1.92	14.96 ± 2.84	1.22 ± 0.31	17.94 ± 3.85
*t*		6.396	29.103	13.785	9.174
*P*		0.000	0.000	0.000	0.000

**Table 3:** Before and after treatment: LTN versus SP in terms of levels (*x* ± *s*, %).

Group	Cases	LTN (pg/ml)		SP (ng/L)	
		Before treatment	After treatment	Before treatment	After treatment
Control group	50	244.64 ± 22.96	265.91 ± 28.96^a^	75.01 ± 7.22	65.91 ± 10.31^a^
Study group	50	244.86 ± 22.75	288.76 ± 28.86^b^	75.05 ± 7.49	54.91 ± 6.91^b^
*t*		0.048	3.951	0.027	6.266
*P*		0.961	0.000	0.978	0.000

*Note.* The control group before and after treatment, ^a^*P* < 0.05; the study group before and after treatment, ^b^*P* < 0.05.

**Table 4:** Comparison of TGF-*β* 1 and TNF-*α* levels between the groups (±*s*).

Group	Cases	TGF-*β*1 (ng/ml)		TNF-*α* (ng/L)	
		Before treatment	After treatment	Before treatment	After treatment
Control group	50	8.59 ± 2.45	9.66 ± 1.67^a^	250.86 ± 25.95	196.92 ± 23.85^a^
Study group	50	8.51 ± 2.53	11.56 ± 1.91^b^	250.64 ± 25.96	125.93 ± 19.85^b^
*t*		0.160	5.295	0.042	16.177
*P*		0.872	0.000	0.966	0.000

*Note*. The control group before and after treatment, ^a^*P* < 0.05; the study group before and after treatment, ^b^*P* < 0.05.

**Table 5:** Comparison of CD3+, CD4+, and CD8+ levels (±*s*, %).

Group	Cases	CD3＋		CD4＋		CD8＋	
		Before treatment	After treatment	Before treatment	After treatment	Before treatment	After treatment
Control group	50	48.83 ± 2.95	51.85 ± 2.91^a^	30.95 ± 1.93	35.96 ± 1.56^a^	37.91 ± 2.94	34.81 ± 2.34^a^
Study group	50	48.93 ± 2.85	58.95 ± 3.91^b^	30.91 ± 1.85	41.94 ± 3.91^b^	37.95 ± 2.81	28.96 ± 3.95^b^
*t*		0.172	10.300	0.105	10.044	0.069	9.010
*P*		0.863	0.000	0.916	0.000	0.944	0.000

*Note*. The control group before and after treatment, ^a^*P* < 0.05; the study group before and after treatment, ^b^*P* < 0.05.

## Data Availability

The datasets used and analyzed during the current study are available from the corresponding author upon reasonable request.

## References

[1] Ni L., Xue P., An C. (2021). Establishment of normal range for thromboelastography in healthy middle-aged and elderly people of weihai in China. *Journal of Healthcare Engineering*.

[2] Zheng L., Feng H., Yin L. (2021). Study on the correlation factors of tumour prognosis after intravascular interventional therapy. *Journal of Healthcare Engineering*.

[3] Matsumoto K., Sakamoto N., Murakami T. (2021). Long-term relapse-free treatment with endoscopic submucosal dissection combined with magnifying narrow-band imaging for a pregnant patient with flat-type condyloma acuminatum: a case report. *Clinical Journal of Gastroenterology*.

[4] Yin G., Li X., Wang X., Zhang H. (2019). Effect of 5-aminolevulinic acid photodynamic therapy on the expression of apoptosis inhibitors Bcl-2 and Survivin in keratinocytes of condyloma acuminatum. *Photodiagnosis and Photodynamic Therapy*.

[5] Xiaomei X., Dong W., Wang B. (2020). Determination of peripheral blood lymphocytes and cytokines in elderly patients with condyloma acuminatum before and after photodynamic therapy. *Chinese Journal of Gerontology*.

[6] Yang Z., Xiong H., Shanshan W. (2019). Yes-associated protein promotes the development of condyloma acuminatum through EGFR pathway activation. *Dermatology*.

[7] Li-Chao L., Hu B., Zhang S.-P. (2019). Reply to “Immune response of condyloma acuminatum after 5-aminolevulinicacid-photodynamic therapy treatment”. *Journal of the Chinese Medical Association : Journal of the Chinese Medical Association*.

[8] Szinai M., Nagy Z., Petra M. (2019). Comparative analysis of human papillomavirus type 6 complete genomes originated from head and neck and anogenital disorders. *Infection, Genetics and Evolution*.

[9] Li-Chao L., Hu B., Zhang S.-P. (2019). Macrophages participate in the immunosuppression of condyloma acuminatum through the PD-1/PD-L1 signaling pathway. *Journal of the Chinese Medical Association : Journal of the Chinese Medical Association*.

[10] Zhang L., Li X., Liu X., Gao Y., Tang Q. (2019). Treatment of multi-position condyloma acuminatum using topical CO 2 laser combined with photodynamic therapy – report of 6 cases[J]. *Photodiagnosis and Photodynamic Therapy*.

[11] Li S., Lu S., Hu R. (2019). Combined treatment of perianal condyloma acuminatum inHIV seropositive men who have sex with men with microwave and photo-dynamic therapy. *Chinese Journal of Experimental and Clinical Virology*.

[12] Fan Z., Wang S., Xu C. (2021). Bioinformatics analysis of differentially expressed genes related to condyloma acuminatum [J/OL]. *Chinese Journal of Dermatology and venereology*.

[13] Dias M. C., Stuqui B., Provazzi P. J. S. (2019). Analysis of nucleotide alterations in the E6 genomic region of human papillomavirus types 6 and 11 in condyloma acuminatum samples from Brazil. *Advances in Virology*.

[14] Zhao Y., Chen Y., Ji S. (2021). Clinical study of carbon dioxide laser combined with 5-aminolevulinic acid photodynamic therapy in the treatment of recurrent condyloma acuminatum. *Journal of Clinical Dermatology*.

[15] Ao C., Xie J., Wang L. (2018). 5-aminolevulinic acid photodynamic therapy for anal canal condyloma acuminatum: a series of 19 cases and literature review. *Photodiagnosis and Photodynamic Therapy*.

[16] Zhong Q., Li K., Chen D., Wang H, Lin Q, Liu W (2018). Rapid detection and subtyping of human papillomaviruses in condyloma acuminatum using loop-mediated isothermal amplification with hydroxynaphthol blue dye. *British Journal of Biomedical Science*.

[17] Furukawa S., Uota S., Yamana T. (2018). Distribution of human papillomavirus genotype in anal condyloma acuminatum among Japanese men: the higher prevalence of high risk human papillomavirus in men who have sex with men with HIV infection. *AIDS Research and Human Retroviruses*.

[18] Guo Y., Liu M., Yu J. (2021). Study on the factors of recurrence of condyloma acuminatum treated with photodynamic therapy alone or in combination with other traditional methods [J/OL]. *Chinese Journal of Dermatology and venereology*.

[19] Zheng Y., Liu X., Feng Y. (2021). HPV infection in perianal tissue of male HIV/AIDS patients with perianal verrucous vegetation [J]. *AIDS and STD in China*.

[20] Sun Y.-Z., Li J.-F., Wei Z.-D. (2019). Proteomic and bioinformatic analysis of condyloma acuminata: mild hyperthermia treatment reveals compromised HPV infectivity of keratinocytes via regulation of metabolism, differentiation and anti-viral responses. *International Journal of Hyperthermia*.

[21] Zhou S., Gu L., Shi Z. (2021). Effect of oral thymic peptide on recurrence rate of condyloma acuminatum treated by CO_2 laser combined with photodynamic therapy. *Chinese Journal of Dermatology and venereology*.

[22] Xie J., Wang S., Li Z. (2019). 5-aminolevulinic acid photodynamic therapy reduces HPV viral load via autophagy and apoptosis by modulating Ras/Raf/MEK/ERK and PI3K/AKT pathways in HeLa cells[J]. *Journal of Photochemistry and Photobiology B: Biology*.

[23] Lang R., Huang T., Zhu D. (2021). Surgery combined with superficial X-ray in the treatment of 1 case of familial benign chronic pemphigus complicated with condyloma acuminatum. *Journal of Clinical Dermatology*.

[24] Meng X., Li Y., Luan H., Shi X (2018). Therapeutic effect of photodynamic therapy combined with imiquimod in the treatment of anal condyloma acuminatum and its effect on immune function. *Experimental and Therapeutic Medicine*.

[25] Li Y., Zeng B., Zheng Z. (2021). Effect of carbon dioxide laser combined with photodynamic therapy on human papillomavirus load in patients with perianal condyloma acuminatum. *Journal of Clinical Dermatology*.

[26] Li Z., Yu X., Hua Y. (2021). Observation on the efficacy of photodynamic therapy with thermosensitive gel as matrix in the treatment of anal condyloma acuminatum. *Journal of Clinical Dermatology*.

[27] Hu Y., Lu Y., Qi X. (2019). Clinical efficacy of paiteling in the treatment of condyloma acuminatum infected with different subtypes of HPV. *Dermatologic Therapy*.

